# Feasibility and Validity of Cambridge Neuropsychological Test Automated Battery in Mild Cognitive Impairment Screening for Patients with Atrial Fibrillation

This article has been retracted.

**DOI:** 10.1155/2022/1527292

**Published:** 2022-02-08

**Authors:** Jia Wang, Yiwei Lai, Chao Jiang, Yu Bai, Baolei Xu, Xin Du, Jianzeng Dong, Changsheng Ma

**Affiliations:** ^1^Department of Cardiology, Beijing Anzhen Hospital, Capital Medical University, National Clinical Research Centre for Cardiovascular Diseases, Beijing Advanced Innovation Center for Big Data-Based Precision Medicine for Cardiovascular Diseases, Beijing, China; ^2^Faculty of Science, The University of Sydney, Sydney, Australia; ^3^Department of Neurology, Beijing Anzhen Hospital, China

## Abstract

**Background:**

Atrial fibrillation (AF) is associated with the worsening of cognitive function. Strategies that are both convenient and reliable for cognitive screening of AF patients remain underdeveloped. We aimed to analyze the sensitivity and specificity of computerized cognitive screening strategies using subtests from Cambridge Neuropsychological Test Automated Battery (CANTAB) in AF patients.

**Methods:**

The Multitasking Test (MTT), Rapid Visual Information Processing (RVP), and Paired Associates Learning (PAL) subtests from CANTAB were performed in 105 AF patients. Traditional standard neuropsychological tests were used as a reference standard. Cognitive screening models using different CANTAB subtests were established using multivariable logistic regression. Further stepwise regression using the Akaike Information Criterion (AIC) was applied to optimize the models. Receiver operating characteristic curve analyses were used to study the sensitivity and specificity of these models.

**Results:**

Fifty-eight (55%) patients were diagnosed with mild cognitive impairment (MCI). MTT alone had reasonable sensitivity (82.8%) and specificity (74.5%) for MCI screening, while RVP (sensitivity 72.4%, specificity 70.2%) and PAL (sensitivity 70.7%, specificity 57.4%) were less effective. Stepwise regression of all available variables revealed that a combination of MTT and RVP brought about higher specificity (sensitivity 82.8%, specificity 85.8%), while PAL was not included in the optimal model. Moreover, adding education to the models did not result in improved validity for MCI screening.

**Conclusion:**

The CANTAB subtests are feasible and effective strategies for MCI screening among AF patients independent of patients' education levels. Hence, they are practical for cardiologists or general practitioners.

## 1. Introduction

Atrial fibrillation (AF) is a significant public health problem due to its increasing mortality rate, higher risks of stroke and heart failure, and escalating health care expenses [1]. In recent years, emerging evidence has revealed a higher risk of cognitive impairment among AF patients [2]. About 22%-51% of AF individuals are undergoing cognitive impairment [3, 4].

Mild cognitive impairment (MCI) is a condition in which individuals demonstrate cognitive decline with or without minimal impairment of instrumental activities of daily living (IADL) [5]. It is a critical stage for early treatment and prevention in the natural history of cognitive decline. However, MCI is often neglected by both physicians and patients for its mild symptoms. In AF patients, the prevalence of MCI could be as high as 60% in previous studies and patients may go through MCI even at a young age [6–8]. As a nonnegligible complication of AF, more emphasis should be placed on mild cognitive impairment and it should be routinely screened in clinical practice. However, our current understanding is limited, as only a few instruments were validated and were able to characterize patterns of cognitive impairment in the AF population. Furthermore, considering the necessity of long-term cognitive monitoring in the AF population, conventional paper-based scales that require in-person interviews and may have practice effect in the long run may not be the best choice.

With the rapid development of societies and economies worldwide, health technologies have been enhanced [9]. The Cambridge Neuropsychological Test Automated Battery (CANTAB) is a computerized neuropsychological test battery [10]. The tests are all standardized by automated voiceover instructions and are simple to use. In the present study, we aim to investigate an automated MCI screening strategy using CANTAB subtests to facilitate clinical management of cognitive impairment in AF patients.

## 2. Methods

### 2.1. Study Design and Population

The present study was approved by the ethics committee of Beijing Anzhen Hospital (D11110700300000) and was conducted ethically in accordance with the World Medical Association Declaration of Helsinki. Chinese-speaking AF patients were randomly enrolled between September 2019 and January 2020 from a tertiary medical center (Beijing Anzhen Hospital, Beijing, China). Inclusion criteria are as follows: (1) complete clinical data, (2) in accordance with the diagnostic criteria of AF (AF was documented by a standard 12-lead electrocardiogram), (3) patient age over 50 years, and (4) no abnormalities in hearing or vision. Exclusion criteria were (1) known neurological or psychiatric disease or dementia, (2) alcoholism (40 mg for males and 20 mg for females) or antipsychotics, (3) patients who cannot or are unable to complete cognitive tests, and (4) patients who were treated with catheter ablation. All 105 patients were able to complete traditional standard neuropsychological tests and CANTAB tests independently and orderly. Demographics and medical histories were extracted from electronic medical records. The flow chart of the study is shown in Figure 1.

### 2.2. Standard Cognitive Assessments and Reference Standard

The standard cognitive assessments used for MCI diagnosis in the present study are comprised of a setting of traditional standard neuropsychological tests with published normative data of the Chinese population. As recommended by the 2018 Chinese guideline for the management of dementia and cognitive disorders [11], we applied the Huashan version of the auditory verbal learning test (AVLT-H) [12] to assess episodic memory; in the auditory verbal learning test (AVLT), there are 12 words from three categories (flowers, occupations, and apparels) with four words for each category in the list. The AVLT-H measures both short-term recall (3- or 5-minute delay) and long-term recall (20-minute delay) of the 12 words in the list over three learning trials. The digit span test (DST) [13] is for attention and working memory; in the test, there is a list of consecutive numbers; in the first trial, participants are asked to recall the consecutive numbers in the same order; in the second trial, participants should recall the numbers in the reverse order. The trail making tests A and B (TMT A and B) [14] are for executive function and information processing speed. In TMT A, the participant is asked to draw a line from 1 through 25 as fast as possible. In TMT B, the numbers are contained in circle and square shapes; the participant is asked to connect the numbers in order from the numbers 1 to 25 as quickly as possible. The semantic and phonetic verbal fluency test (VFT) [13] is for language; it consisted of two parts: phonetic verbal fluency test and semantic verbal fluency test. The phonetic verbal fluency test asked subjects to recall as many words beginning with “yi” and “wan” as they could in 2 minutes; the score is the total number of “yi” and “wan.” The semantic verbal fluency test requires the participant to generate words from the category of animals and commodities; every participant is told to name animals for 60 s. The score is the total number of animals and the commodities in 1 min. And the Rey-Osterrieth complex figure test (RCFT) [15] is for visual spatial ability; the participants were required to imitate the graph and recall the graph about 20 minutes later without being reminded. The total score was 36 points. Besides, the functional activity questionnaire (FAQ) [16] was evaluated in all patients. All abovementioned tests were administered by the same physician (J Wang) who had been trained for these tests to ensure test quality consistency across all patients.

The reference standard for MCI using Jak/Bondi criteria [17] is (1) impairment in any one of the cognitive tests (defined as >1.5 SD below the age-corrected normative mean) and (2) normal or mildly impaired daily activity (FAQ < 9).

### 2.3. Cambridge Automatic Neuropsychological Test Battery (CANTAB) Subtests

The CANTAB is a computerized cognitive test battery originally developed for the elderly population, containing 25 subtests for 7 cognitive domains. Considering that memory [18], attention [19], and executive function [20, 21] are most commonly impaired in AF patients, three corresponding subtests were selected in the present study.

1. Multitasking Test (MTT) [22] is a test of executive function which provides a measure of the ability to use multiple sources of potentially conflicting information to guide behavior; it can be done in 8 minutes. During each trial, an arrow appears on the right or left side of the screen, and the subject will be asked to make a right or left response. Before each trial, instructions on whether to respond according to “direction” or “side” will be provided to the subject. For sections of the test, the arrows' directions and sides are incongruent
2. Rapid Visual Information Processing (RVP) [23] is a sensitive tool to assess sustained attention and processing speed; it can be done in 9 minutes. In the test, there will be a white box in the center of the screen; single digits from 2 to 9 will appear in pseudorandom order at a rate of 100 digits per minute. Subjects must detect the target sequences (3-5-7) and press the button as a response
3. Paired Associates Learning (PAL) [23] is a sensitive tool to assess episodic memory and new learning; it can be done in 8 minutes. In the test, boxes will be opened on the screen in a randomized order to display the patterns hidden inside. The patterns will appear in the center of the screen, one at a time, and the subjects must touch the box where the pattern was originally located

The patients completed the CANTAB subtests using an iPad under the voiceover instructions of the system without any help from physicians. The test results were generated automatically by the testing system.

### 2.4. Statistical Analysis

R 3.5.1 was used for data analyses. We calculated the differences in test scores between MCI and cognitively normal patients using *χ*^2^ or *t*-tests. Pearson or Spearman correlation analyses were then conducted to examine the association between CANTAB models and the standard tests.

Model generation was conducted in a computerized method. Each CANTAB subtest provides a quantity of variables to describe cognitive function. Variables of each subtest together with age and education level were included in a multivariate logistic model, and stepwise regression was conducted to optimize the models (Table 1). The stepwise regression conformed to the Akaike Information Criterion (AIC) and was achieved by the “stepAIC” function in the R package “MASS.” Likewise, age, education level, and all available variables from all three subtests were included in one logistic model and then optimized in the same way to investigate the most effective and efficient combination of subtests.

Receiver operating characteristic (ROC) curve analyses were further conducted to determine and compare the validity of each model, using the pROC package [24]. Among all cut-off points, the cut-off point with the highest Yourdon index (sensitivity > 80%) is selected as the optimal threshold of the model. Considering the clinical importance of education in cognitive assessment, education was included in all CANTAB models for sensitivity analysis.

Sample size estimation is conducted by PASS 15.0. 45 cases have 0.9 power to validate a sensitivity of 80%, under the null hypothesis of sensitivity = 60%. Assuming the prevalence of MCI is 30% to 50% in the present study, at least 90 patients should be enrolled.

## 3. Results

### 3.1. Demographics of Study Population

Baseline characteristics of all included individuals are shown in Table 2. The population studied has an average age of 63.8; 70 (66.7%) of them were male. 61 (58.1%) of the patients had 7-12 years of education, while 24 (22.9%) had >12 years of education and 20 (19.0%) had ≤6 years of education. Hypertension is the most common comorbidity occurring in 64 (61.0%) patients, followed by dyslipidemia (32.4%) and diabetes (21.9%). Eight (7.6%) patients had a history of stroke. All patients were given oral anticoagulants because of the radiofrequency ablation.

### 3.2. Distribution of Cognition in Atrial Fibrillation Patients

According to the standard neuropsychological assessment (five cognitive domain tests), 47 patients were cognitively normal, and 58 patients had mild cognitive impairment. Of the 105 AF patients, 27.0% indicated single domain cognitive impairment, 28.0% had multidomain cognitive impairment. 47 (81.0%) of the MCI were nonamnestic, while only 2 (3.4%) were single-domain amnestic MCI. The detailed distribution of impaired cognitive domain in MCI with AF is shown in Figure 2. Among patients with MCI, executive function was most commonly impaired (*n* = 38), followed by attention (*n* = 27), visual spatial function (*n* = 21), memory (*n* = 11), and language (*n* = 8).

### 3.3. Performance of CANTAB Models in MCI Screening

The models created by stepwise regression using single or multiple CANTAB subtests and their optimal sensitivity and specificity are listed in Table 3, and the ROC curves are shown in Figure 3. For a single CANTAB subtest, MTT alone could reach both reasonable sensitivity (82.8%) and specificity (74.5%) for MCI screening independent of age and education level, while the validities of models using RVP (sensitivity = 72.4%, specificity = 70.2%) or PAL (sensitivity = 70.7%, specificity = 57.4%) were inadequate as an ideal screening tool. After stepwise regression of age, education level and all available variables from the three tests, age, and variables from MTT and RVP were included in the optimal model (model 4), which had the same sensitivity (82.8%) as model 3 but resulted in higher specificity (85.1%). Education level as an additional factor to the models failed to improve the optimal sensitivity or specificity, further verifying the reliability and stability of the models (Table 4).

### 3.4. Correlation between CANTAB Models and Standard Cognitive Tests

Correlations between computerized models and traditional battery are shown in Table 5. The models representing PAL (model 1), RVP (model 2), MTT (model 3), and a combination of CANTAB tests (model 4) were significantly correlated with all standard tests to different extents; model 3 and model 4 showed a better correlation in all cognitive domains.

## 4. Discussion

AF plays a significant role in cognitive decline. Emerging evidence highlighted the possibility of AF patients going through cognitive decline at a younger age [8]. Several studies have also demonstrated the negative impacts of MCI on the prognosis and treatment of AF patients [25, 26]. For example, AF patients with MCI may have to undergo worse anticoagulant compliance and poorer international normalized ratio (INR) control [25]. MCI may also influence AF patients' ability to self-care and perform daily work [25]; the AF patients with MCI had low gait speed which impaired their quality of life [26]. Therefore, cognitive screening for MCI is crucial for AF patients to identify cognitive impairment at an early stage so that immediate preventative measures such as lifestyle improvement and cognitive training can be taken. Preservation of mental health may in turn favour medication compliance and management of AF. Hence, cognitive screening should be a routine consideration in the clinical management of AF.

Executive function is more vulnerable in AF patients than general populations [19]; this implies the importance of MTT in MCI screening of AF patients. The correlation of MTT and RVP to cognitive domains other than executive function and attention provides these tests with additional feasibility and efficacy. A combination of MTT and RVP results in higher specificity than MTT alone, but at the cost of longer testing time (8 minutes vs. 17 minutes). Therefore, clinical application should be at the discretion of clinical circumstances; RVP should be considered if more misdiagnoses were to be avoided.

It is well established that limited education or schooling is associated with cognitive decline [27–30]. Cognitive assessment of these older adults is particularly challenging, because the comprehension of some traditional texts requires a certain level of education [31]. Intriguingly, in the present study, education is automatically excluded by stepwise regression in all the models; the sensitivity analysis indicated that it provides no extra increase in sensitivity and specificity regardless of the component of the models. This result is consistent with previous findings [32], indicating that CANTAB can be widely applied in patients with varying education levels without needing to adjust the model for differing education backgrounds of patients.

In the present study, the screening strategy based on CANTAB is studied expressly in the AF population, which may outperform the conventional clinical practice where scales originated from the geriatric or Alzheimer population were applied. Montreal cognitive assessment (MoCA) is the most commonly used instrument in MCI screening, but the results of MoCA can be affected by many factors, such as cultural background, education level, and the neurological physicians or professional researchers conducting the assessment. Although the sensitivity of the CANTAB strategy for the AF population is comparable to the sensitivity of MoCA for the general population [33], the CANTAB strategy may be advantageous in many aspects. The CANTAB tests not only have a short testing time but also reduce the burden of test administration such as recording, scoring, and training of the administrators [34]. More importantly, unlike MoCA or the paper-pencil tests, CANTAB can minimize the practice effects, which occurs as a result of repeated testing, leading to an overestimation of the treatment effects and an underestimation of the disease progression [34, 35]. In addition, the predominantly nonverbal nature of the tests minimizes the risk of errors arising from differences in language or cultural understanding. As a remote cognitive screening tool, CANTAB prevents the problem of failing to complete follow-ups. Thus, CANTAB is an ideal instrument in longitudinal studies to trace the decline of cognitive functions.

The present study has several limitations. Firstly, The number of cases we can collect is not many. And selection bias may occur, as some patients refused the neuropsychological testing. Meanwhile, the CANTAB tests are less feasible in patients with hearing loss who are at high risk of cognitive impairment. Secondly, we did not evaluate the visual-spatial ability test and language function. Whether implementation of these subtests can lead to an additional increase in screening validity requires further study, though at the cost of prolonged testing time.

## 5. Conclusion

In conclusion, the CANTAB subtests are feasible and effective in identifying MCI patients in the AF population. It is an ideal preliminary screening instrument for cardiologists or general practitioners, because it is effective and simple to navigate. And it may further facilitate timely intervention and the preservation of mental health in AF patients.

## Figures and Tables

**Figure 1:** Flowchart of patients' selection.

**Figure 2:** Distribution of cognitive domain impairment in MCI with atrial fibrillation patients.

**Figure 3:** The ROC curves for MCI screening models using CANTAB subtests.

**Table 1:** The annotation for each model classification.

Types of models	Classification criteria
Model 1	Age, PALTEA
Model 2	Age, RVPA, RVPLSD, RVPML
Model 3	Age, MTTTIC, MTTLMD, MTTMTCMD
Model 4	Age, RVPA, RVPML, MTTTIC, MTTLMD, MTTMTCMD
Model 1′	Age, education, PALTEA
Model 2′	Age, education, RVPA, RVPLSD, RVPML
Model 3′	Age, education, MTTTIC, MTTLMD, MTTMTCMD
Model 4′	Age, education, RVPA, RVPML, MTTTIC, MTTLMD, MTTMTCMD

**Table 2:** Characteristics of the study population.

Variables	All of the AF patients (*n* = 105)
Age (years)	63.8 ± 6.3
≥75	8 (7.6%)
65-74	34 (32.4%)
<65	63 (60.0%)
Sex	
Male	70 (66.7%)
Female	35 (33.3%)
SBP (mmHg)	126 ± 14
Education (years)	10.1 ± 4.0
≤6	20 (19.0%)
7-12	61 (58.1%)
>12	24 (22.9%)
Smoking (%)	
Yes	13 (12.4%)
No	92 (87.6%)
eGFR < 60 mL/min/1.73 m^2^ (%)	5 (4.8%)
Hypertension (%)	
Yes	64 (61.0%)
No	41 (39.0%)
Diabetes (%)	
Yes	23 (21.9%)
No	82 (78.1%)
Dyslipidemia (%)	
Yes	34 (32.4%)
No	71 (67.6%)
Stroke (%)	
Yes	8 (7.6%)
No	97 (92.4%)
Heart failure (%)	
Yes	8 (7.6%)
No	97 (92.4%)
Coronary heart disease (%)	
Yes	13 (12.4%)
No	92 (87.6%)
Anticoagulant drugs	105 (100%)

SBP: systolic blood pressure; eGFR: estimated glomerular filtration rate.

**Table 3:** Computerized models, the cut-off, and parameters' *β* value.

Models	AUC (95% CI)	Sensitivity	Specificity	Cut-off	Parameter	*β*
Model 1	0.667 (0.563-0.770)	70.7%	57.4%	0.522	Age PALTEA Intercept	-0.0107 0.0091 0.9287
Model 2	0.783 (0.695-0.870)	72.4%	70.2%	0.539	Age RVPA RVPLSD RVPML Intercept	-0.0193 -3.1215 0.0018 0.0023 3.5757
Model 3	0.846 (0.77-0.923)	82.8%	74.5%	0.520	Age MTTTIC MTTLMD MTTMTCMD Intercept	-0.0550 0.0078 0.0013 -0.0006 -0.5180
Model 4	0.875 (0.806-0.945)	82.8%	85.1%	0.515	Age RVPA RVPML MTTTIC MTTLMD MTTMTCMD Intercept	-0.0152 -3.3253 0.0016 0.0046 0.0013 -0.0005 2.9646

PALTEA: PAL total errors (adjusted), the number of times the subject chose the incorrect box for a stimulus on assessment problems. RVPA: RVPA′, A′ (A prime) is the signal detection measure of a subject's sensitivity to the target sequence (string of three numbers), regardless of response tendency (the expected range is 0.00 to 1.00; bad to good). RVPML: RVP mean response latency, the mean response latency on trials where the subject responded correctly. Calculated across all assessed trials. RVPLSD: RVP response latency (SD), the standard deviation of response latency on trials where the subject responded correctly. MTTTIC: MTT total incorrect, the number of trials for which the outcome was an incorrect response (subject pressed the incorrect button within the response window). Calculated across all assessed trials. MTTLMD: MTT reaction latency (median), the median latency of response (from stimulus appearance to button press). Calculated across all correct, assessed trials. MTTMTCMD: MTT multitasking cost (median), the difference between the median latency of response (from stimulus appearance to button press) during assessed blocks in which both rules are used versus assessed blocks in which only a single rule is used. Calculated by subtracting the median latency of response during single-task block(s) from the median latency of response during multitasking block(s).

**Table 4:** Computerized models with education.

Models	AUC (95% CI)	Sensitivity	Specificity
Model 1′	0.677 (0.575-0.779)	75.9%	48.9%
Model 2′	0.785 (0.698-0.872)	72.4%	70.2%
Model 3′	0.858 (0.786-0.931)	82.8%	70.2%
Model 4′	0.879 (0.809-0.948)	82.8%	87.2%

**Table 5:** Correlations between models and standard neuropsychological tests.

Models	AVLT-H (short time delay)		AVLT-H (long time delay)		Rey-Osterrieth		TMT A		TMT B		DST		VFT	
	*r*	*p*	*r*	*p*	*r*	*p*	*r*	*p*	*r*	*p*	*r*	*p*	*r*	*p*
Model 1	-0.398	<0.001	-0.479	<0.001	-0.369	<0.001	0.289	0.003	0.285	0.003	-0.208	0.033	-0.226	0.021
Model 2	-0.256	0.008	-0.304	0.002	-0.334	<0.001	0.538	<0.001	0.390	<0.001	-0.341	<0.001	-0.405	<0.001
Model 3	-0.363	<0.001	-0.403	<0.001	-0.401	<0.001	0.523	<0.001	0.531	<0.001	-0.544	<0.001	-0.382	<0.001
Model 4	-0.346	<0.001	-0.405	<0.001	-0.419	<0.001	0.602	<0.001	0.538	<0.001	-0.506	<0.001	-0.445	<0.001

## Data Availability

The data used to support the findings of this study are available from the corresponding authors upon request.
